# Continuous Lumbar Plexus Block under the Guidance of the “Shamrock Method” Ultrasound: Analgesic Effects and Hemodynamic Effects after Total Knee Arthroplasty in Elderly Patients

**DOI:** 10.1155/2021/3531236

**Published:** 2021-10-18

**Authors:** Jinpei Xue, Xiang Fu, Zurong Hu

**Affiliations:** ^1^Department of Anesthesiology, Longgang Orthopaedics Hospital of Shenzhen, Shenzhen, Guangdong 518112, China; ^2^Department of Anesthesiology, Guangdong Women and Children Hospital, Guangzhou, Guangdong 510010, China

## Abstract

**Objective:**

To explore the effect of continuous lumbar plexus block guided by the “Shamrock method” on postoperative analgesia and hemodynamics in elderly patients after total knee arthroplasty (TKA).

**Methods:**

From January 2020 to December 2020 in our hospital, 98 patients who underwent TKA were selected. Using the random number table method, the patients were divided into two groups: a continuous lumbar plexus block group (group L), with 49 patients, and a continuous femoral nerve block group (group F), with 49 patients. The onset time and maintenance time of motor and sensory nerve blocks in patients were recorded. A visual analogue scale (VAS) was applied to assess the pain severity at 6, 12, 24, and 48 h after the operation. The VAS score (FVAS) was applied to evaluate the pain severity of the patients during 24 and 48 h after the operation and knee joint functional exercise. The levels of hemodynamic indexes such as heart rate, mean arterial pressure, and oxyhemoglobin saturation and the levels of hemorheological indexes such as plasma viscosity, high and low whole blood shear viscosity, fibrinogen, and hematocrit were detected and compared between the two groups immediately after the operation and at 12 h and 48 h after the operation, respectively. The incidence of adverse reactions induced by anesthesia was counted.

**Results:**

The onset time of motor and sensory nerve blocks in group L was lower than that in group F, and the maintenance time was higher than that in group F (*P* < 0.05). The VAS scores of 6, 12, 24, and 48 h after operation in group L were significantly lower than those in group F (*P* < 0.05). The FVAS scores of group L at 24 and 48 h after operation were significantly lower than those of group F (*P* < 0.05). The heart rates of the patients in the two groups were higher at 12 h and 48 h after operation than those immediately after operation (*P* < 0.05). The heart rates at 12 h and 48 h after operation in group L were lower than those in group F (*P* < 0.05). The plasma viscosity, high whole blood shear viscosity, and low whole blood shear viscosity in the group L at 12 h and 48 h after operation were lower than those in group F (*P* < 0.05). There was no significant difference in the incidence of local anesthetic poisoning, nausea, vomiting, urinary retention, pruritus, and other adverse reactions between the two groups (*P* > 0.05).

**Conclusion:**

The “Shamrock method” ultrasound-guided continuous lumbar plexus block in elderly patients after TKA has good analgesic effect, stable hemodynamics, little influence on hemorheology, and good safety. It is of great value to enhance the surgical effect and promote postoperative rehabilitation.

## 1. Introduction

With the aging of the population, degenerative diseases of joints are also increasing. Total knee arthroplasty (TKA) is a major technique for the treatment of severe knee joint disorders and the reconstruction of knee function, which can relieve knee pain and reconstruct knee function [1]. However, TKA is traumatic, and the patient's stress response is great, which often leads to severe postoperative pain, thus affecting the recovery of patients to some extent. Therefore, it is necessary to select an appropriate postoperative analgesic method [2]. Because of spinal degeneration and other reasons, there are many difficulties in anesthesia puncture in elderly patients. In addition, changing the posture when anesthesia is performed and controlling the dosage of anesthetics and anesthesia level during the operation are required, which are likely to affect the hemodynamic stability of patients to a certain extent. In particular, elderly patients are often accompanied by systemic medical diseases which increase the anesthesia risk and limit its clinical application [3]. Ultrasound guidance is beneficial for the localization of nerve blocks and can ensure the full diffusion of local anesthetics into the target nerve area. Thereby, it reduces puncture complications. Ultrasound-guided continuous femoral nerve block for postoperative analgesia is widely used in clinical practice. However, due to incomplete obturator nerve block and incomplete puncture in the ultrasound image, it is difficult to control the depth of the needle insertion and often difficult to achieve a satisfactory analgesic effect [4, 5]. The “Shamrock method” is a new ultrasonic-guided lumbar plexus nerve block method with in-plane needle insertion, in which a low-frequency probe is placed at the head side of the iliac crest of a patient to obtain ultrasound cross-sectional images of the lumbar spine and paravertebral structure, including ultrasound images of the lumbar plexus nerve. From ultrasound images, the diffusion of a local anesthetic around the nerve was observed in real time. Compared with nerve stimulator localization, ultrasound-guided localization has obvious advantages. Ultrasound-guided positioning has obvious advantages over nerve stimulator positioning. Under ultrasound guidance, the relationship between the needle and nerves as well as the surrounding vascular tissues can be directly observed and the success rate of block is improved, thus reducing the occurrence of complications such as kidney and nerve damage [6, 7]. In this study, the “Shamrock method” was used to guide continuous lumbar plexus block and continuous femoral nerve block and to compare the analgesic effects and hemodynamic effects of the two ways on elderly patients after TKA.

## 2. Materials and Methods

### 2.1. General Information

From January 2020 to December 2020, 98 patients (41 males and 57 females), aged 60–75 years and weighing 45–98 kg, were classified as classes II–III by the American Association of Anesthesiologists (ASA) and underwent TKA in our hospital. Inclusion criteria are as follows: no previous history of local anesthesia drug allergy or opioid addiction; no peripheral neuropathy and coagulation disorders; and no contraindication for peripheral nerve block. Exclusion criteria are as follows: patients complicated by severe liver and kidney failure after preoperative examination; patients allergic to narcotic drugs or postoperative analgesic drugs; patients with a history of neuropsychiatric disease or stroke; patients who are chronic alcoholic; patients with unclear consciousness and unable to cooperate with postoperative functional exercise; and patients on steroids or opioids.

Using the random number table method, the patients were divided into two groups: a continuous lumbar plexus block group (group L), with 49 patients, and a continuous femoral nerve block group (group F), with 49 patients. This study was reviewed and approved by the Hospital Ethics Committee, and all patients provided informed consent.

### 2.2. Anesthesia Method

After entering the operation room, the venous channels were opened in both groups, and noninvasive blood pressure, heart rate, ECG, and pulse oximetry were routinely monitored with multifunctional monitors. A nerve block was performed 30 min before the operation, and midazolam 1-2 mg and fentanyl 50 *μ*g were intravenously injected before anesthesia.

The patients in group L were treated with continuous lumbar plexus block under the localization of the “Shamrock method” ultrasound guidance combined with a stimulator. The patient was laid in the lateral decubitus position, and the affected side was on the upper limb. The lower limbs stretched naturally and flexed slightly, taking the line connecting the spinous processes of the spine as the midline and the highest point of the iliac crest as the perpendicular line intersecting with the abovementioned line. The transverse movement of the abdominal muscle aponeurosis was located as quadratus lumborum. Quadratus lumborum is inserted at the top of the L_1–4_ transverse process, and ultrasound could identify the L_4_ transverse process and the L_4_ vertebral body. The psoas major muscle was located on the ventral side of the transverse process, the erector spinae was located on the dorsal side of the transverse process, and the quadratus lumborum was located on the tip of the L_4_ transverse process. The L_4_ transverse process was taken as the center of these three muscles to form an easily identifiable “clover” structure. The puncture point was located 4–5 cm from the intersection point of the two straight lines to the side of the block. After the puncture point was determined, a low-frequency linear ultrasonic probe (frequency 2–5 MHz) was used to place the probe laterally on the anterolateral side of the axillary midline, near the high point of the iliac crest. The puncture needle was inserted in an in-plane mode, and the insertion direction was perpendicular to the skin or slightly toward the midline.

In group F, the descending femoral nerve block was located using ultrasound guidance combined with a stimulator. A high-frequency linear array probe (at a frequency of 7–13 MHz) was placed horizontally 2 cm below the inguinal ligament, with the long axis perpendicular to the longitudinal axis of the thigh. After the transverse ultrasound images of the femoral vein, femoral artery, and femoral nerve arranged from inside to outside at the fascia of the iliopubic arch were clearly displayed, the needle was inserted through the skin of the lateral thigh using the in-plane technique. The two groups simultaneously and jointly used a nerve stimulator for auxiliary positioning and the stimulation wave width was set to be 0.1 ms, the frequency to be 2 Hz, and the current intensity to be 1 mA. When quadriceps femoris contraction accompanied by patellar pulsation occurred, the stimulation intensity was reduced and the position of the puncture needle was adjusted. When the current was reduced to 0.3–0.4 mA, the muscle group convulsion still existed and the muscle twitch disappeared after 1 mL of medicine was injected after blood withdrawal and no more. After the stimulation intensity was increased to 1 mA, 30 mL of local anesthetic and 0.2% ropivacaine was continuously injected without muscle contraction. A catheter was retained for 5 cm beyond the needle tip.

All patients were intubated with laryngeal mask airway after nerve block. Intravenous target-controlled infusions of propofol (2.5–3.0 mg/L), fentanyl (50–100 g), and cisatracurium besylate (0.1–0.2 mg/kg) were performed. One-time Supreme laryngeal mask airway (LMA, Germany) was used for intubation. During the operation, 0.6%–1.0% sevoflurane was inhaled, followed by an intravenous target-controlled infusion of 0.8–1.8 mg/L propofol and 0.1–0.2 g/(kg·h) remifentanil to maintain anesthesia and end-tidal partial pressure of carbon dioxide of 35–40 mmHg. The laryngeal mask airway was removed after patients were fully awake after the operation. Before the end of the operation, all patients in the two groups were connected with a one-time postoperative analgesia pump, with the background dose of 0.2% ropivacaine 5 mL/h, and retained for analgesia for 48 h. At any time point when the patient's visual analogue scale (VAS) score was greater than 4, an additional 40 mg of parecoxib sodium was administered intravenously.

### 2.3. Observation Indicators

1. A nerve stimulator was used to record the onset time (from the time the ultrasonic probe was placed on the skin to the time of anesthesia onset) and maintenance time (from the time the anesthesia onset to the time of completing the operation) of motor and sensory nerve blocks in patients.
2. The VAS score was used to evaluate the pain severity at 6, 12, 24, and 48 h after the operation. The VAS score (FVAS) was applied to evaluate the pain severity of the patients during 24 and 48 h after the operation and knee joint functional exercise. The total score was 0–10. The higher the score was, the more severe the pain would be.
3. The levels of hemodynamic indexes such as heart rate, mean arterial pressure, and oxyhemoglobin saturation were detected and compared between the two groups immediately after operation and 12 h and 48 h after the operation, respectively.
4. The plasma viscosity, high and low whole blood shear viscosity, fibrinogen, hematocrit, and other blood rheology indexes were measured immediately after operation and 12 h and 48 h after the operation using the Vital Vedo FASCO-3010B automatic blood flow detector.
5. The incidence of adverse reactions induced by anesthesia was counted.

## 3. Statistical Method

All data were analyzed by using SPSS22.0 statistical software, and measurement data were expressed as mean standard deviation. The independent sample *t*-test was used for pairwise comparison, and repeated measures analysis of variance was used for comparison at different time points. The count data were expressed as the rate (%) using the *χ*^2^ test. *P* < 0.05 indicated that the difference was statistically significant.

## 4. Results

### 4.1. Comparison of General Data between the Two Groups

There was no significant difference in general information such as gender, age, weight, and ASA classification between the two groups (*P* > 0.05), as shown in Table 1.

### 4.2. Comparison of Nerve Block between the Two Groups

The onset time of motor and sensory nerve blocks in group L was lower than that in group F and the maintenance time was higher than that in group F (*P* < 0.05), as shown in Figure 1.

### 4.3. Comparison of the VAS Scores at 6, 12, 24, and 48 h after the Operation between the Two Groups

The VAS scores at 6, 12, 24, and 48 h after the operation in group L were significantly lower than those of group F and the differences were statistically significant (*P* < 0.05), as shown in Figure 2.

### 4.4. Comparison of the FVAS Scores after Functional Exercise at 24 h and 48 h after the Operation between the Two Groups

The FVAS scores of group L at 24 and 48 h after operation were significantly lower than those of group F and the differences were statistically significant (*P* < 0.05), as shown in Figure 3.

### 4.5. Comparison of Hemodynamics Immediately after the Operation and at 12 h and 48 h after the Operation between the Two Groups

The heart rates of the patients in the two groups were higher at 12 h and 48 h after the operation than those immediately after the operation (*P* < 0.05). There were no significant changes in the mean arterial pressure and oxyhemoglobin saturation levels of the patients in the two groups immediately after the operation and at 12 h and 48 h after the operation (*P* > 0.05). The heart rates at 12 h and 48 h after the operation in group L were lower than those in group F and the differences were statistically significant (*P* < 0.05), as shown in Figure 4.

### 4.6. Comparison of Blood Rheology Immediately after the Operation and at 12 h and 48 h after the Operation between the Two Groups

There was no significant difference in plasma viscosity, high whole blood shear viscosity, low whole blood shear viscosity, red blood cell backlog, and fibrinogen between the two groups immediately after the operation (*P* > 0.05). The plasma viscosity, high whole blood shear viscosity, and low whole blood shear viscosity of group L at 12 h and 48 h after the operation were lower than those of group F and the differences were statistically significant (*P* < 0.05), as shown in Figure 5.

### 4.7. Adverse Reactions between the Two Groups

There was no significant difference in the incidence of local anesthetic poisoning, nausea, vomiting, urinary retention, pruritus, and other adverse reactions between the two groups (*P* > 0.05), as shown in Figure 6.

## 5. Discussion

At present, the majority of patients treated with TKA are aged ≥60 years. The physiological function of the elderly has its particularity and low functioning. Combined with complex systemic diseases such as hypertension, diabetes, coronary heart disease, asthma, and other medical complications, postoperative pain often induces a severe stress response, increases the metabolism of patients, and leads to the blood in a hypercoagulable state, which in turn affects the immune function and cardiopulmonary function of patients, especially the elderly patients, which brings challenges to the implementation of anesthesia and perioperative management [8–10].

Peripheral nerve block has obvious disadvantages in elderly patients with blood coagulation dysfunction, many complications, and unstable circulation. Lumbar plexus block, also known as psoas major groove block, is the fascia layer after a local anesthetic is injected into the psoas major muscle. With the development of ultrasound technology, compared with the nerve block assisted by a nerve stimulator, the lumbar plexus nerve block guided by ultrasound allows the visualization of the whole process and can clearly display the specific conditions of the catheter, the puncture needle position, and drug diffusion, not only improving the success rate of the one-time block but also avoiding the vascular damage and nerve damage caused by repeated puncture and reducing the risks of intranerve injection, kidney injury, retroperitoneal hematoma, and intravascular injection. However, due to the deep location of the lumbar plexus, it is difficult to obtain ultrasound anatomical images and the technology is highly dependent, which requires an experienced anesthesiologist to complete it [11, 12].

In this study, the onset time of motor and sensory nerve blocks in group L was lower than that in group F and the maintenance time was higher than that in group F. Besides, the VAS score after the operation was significantly lower than that in group F. It indicated that after continuous injection of drugs for lumbar plexus block under the guidance of the “Shamrock method,” the diffusion process of local anesthetic liquid was significantly shortened and the effect on the obturator nerve was relatively perfect. The liquid was easily diffused to the nerve to generate the blocking effect, which significantly shortened the onset time of the block and improved the analgesic effect. In the study carried out by Nielsen et al. [13], it was pointed out that compared with other techniques, the “Shamrock approach” is considered to be faster and easier to implement and may be safer in terms of potential complications. The needle track and needle tip position just on the side of the lumbar plexus may reduce the risk of adverse reactions and complications.

After reviewing the surgical procedures and summarizing the surgical experience, we considered that intraneural injection could be avoided by observing the needle tip close to the lumbar plexus nerve, connecting the nerve stimulator to educe the patellar tendon beating, and adjusting the appropriate current (the target muscle contraction could be educed when the threshold was within 0.3–0.5 mA). When it could be seen that the needle tip was close to the target nerve and the minimum effective current leading to the contraction of quadriceps femoris was in the range of 0.3–0.5 mA, the position of the needle tip was in the correct position. At the same time, doctors can reduce the distance between the needle insertion point and the target nerve by pressurizing the probe, which makes the operation easier. In addition, by tilting the probe to the head side, we could see an oval structure that rose or fell with the respiration, that is, the ultrasound image of the lower pole of the kidney, to prevent the occurrence of adverse events such as kidney puncture.

The majority of elderly patients receiving TKA often suffer from cardiovascular and cerebrovascular diseases, and the need to maintain hemodynamic stability during anesthesia limits the use of some anesthesia-analgesia methods. On the other hand, in elderly patients, lumbar vertebrae are degenerated to varying degrees, and intervertebral space stenosis and hypertrophy and calcification (ossification) of the ligamentum flavum all cause puncture difficulties to varying degrees. Second, in the implementation of anesthesia, the lateral decubitus position is required. Patients with lower limb injuries of different degrees, especially those with cardiovascular diseases, are prone to hemodynamic changes during the process of postural positioning, which limits their clinical application. For elderly patients, the implementation of anesthesia and perioperative management should not only meet the needs of the operation but also reduce their impact on the physiological function as much as possible, which is conducive to the early postoperative rehabilitation training [14–16]. The results of this study showed that the heart rate of patients in group L was lower than that in group F at 12 h and 48 h after the operation, and the plasma viscosity and high and low whole blood shear viscosity of patients in group L were lower than those in group F at 12 h and 48 h after the operation. These results indicated that continuous lumbar plexus block under the guidance of the “Shamrock method” was better for the postoperative hemodynamic stability than femoral nerve block and the hemorheology of patients was less affected.

Traditional ultrasound-guided lumbar plexus block at the L3 level identifies the lumbar plexus nerve and its surrounding structures using parasagittal and transverse scanning techniques. The needle insertion point is located inside the probe using the in-plane technique. Because of the deep position of the target nerve, low resolution of the low-frequency probe image, and difficulty in identifying the surrounding marker structures, the operation is usually difficult [17]. Compared with the traditional ultrasound-guided lumbar plexus block, the ultrasound anatomical images of the “Shamrock method” lumbar plexus block are more typical, which are closely related to the surrounding tissues and structures for easy recognition. At the same time, the operator can also reduce the distance between the needle insertion point and the target nerve by pressurizing the probe so that the operation is simpler. In addition, by tilting the probe to the head side, we could see an oval structure that rose or fell with the respiration, that is, the ultrasound image of the lower pole of the kidney, to prevent the occurrence of adverse events such as kidney puncture [18–20]. This study showed that there was no statistically significant difference in the incidence of adverse reactions such as local anesthetic poisoning, nausea, vomiting, urinary retention, and pruritus between the two groups. These results show that continuous lumbar plexus block under the guidance of the “Shamrock method” was safe, and at the same time, it ensures the postoperative analgesic effects.

In summary, continuous lumbar plexus block guided by the “Shamrock method” has a good analgesic effect on elderly patients after TKA, with stable hemodynamics, little influence on hemorheology, and good safety. It is of great value to enhance the surgical effect and promote postoperative rehabilitation.

## Figures and Tables

**Figure 1:** Comparison of nerve block between the two groups. *Note.* Compared with the group L, ^*∗*^*P* < 0.05.

**Figure 2:** Comparison of the VAS scores of 6, 12, 24, and 48 h after the operation between the two groups. *Note.* Compared with the group L, ^*∗*^*P* < 0.05.

**Figure 3:** Comparison of the FVAS scores after functional exercise at 24 h and 48 h after operation between the two groups. *Note.* Compared with the group L, ^*∗*^*P* < 0.05.

**Figure 4:** Comparison of hemodynamics immediately after operation and at 12 h and 48 h after operation between the two groups. *Note.* Compared with immediately after operation, ^*∗*^*P* < 0.05 and compared with the group L, ^#^*P* < 0.05.

**Figure 5:** Comparison of blood rheology immediately after operation and at 12 h and 48 h after operation between the two groups. *Note.* Compared with the group L, ^*∗*^*P* < 0.05.

**Figure 6:** Adverse reactions between the two groups.

**Table 1:** Comparison of general data between the two groups.

Group	Male/female	Age (years)	Body weight (kg)	ASA II/III
Group L (*n* = 49)	20/29	65.24 ± 5.19	62.84 ± 6.35	32/17
Group F (*n* = 49)	21/28	66.43 ± 5.37	63.19 ± 7.11	35/14
*t*/*χ*^2^ value	0.042	0.110	0.257	0.425
*P* value	0.838	0.912	0.798	0.515

## Data Availability

The data can be obtained from the corresponding author upon reasonable request.
